RETRACTED

# Five Active Components Compatibility of Astragali Radix and Angelicae Sinensis Radix Protect Hematopoietic Function Against Cyclophosphamide-Induced Injury in Mice and t-BHP–Induced Injury in HSCs

**DOI:** 10.3389/fphar.2019.00936

**Published:** 2019-08-22

**Authors:** Wei Zhang, Jia-huan Zhu, Hao Xu, Xiao-Ping Huang, Xiao-Dan Liu, Chang-Qing Deng

**Affiliations:** ^1^Key Laboratory of Hunan Province for Integrated Traditional Chinese and Western Medicine on Prevention and Treatment of Cardio-Cerebral Diseases, Hunan University of Chinese Medicine, Changsha, China; ^2^Key Laboratory of Colleges and Universities in Hunan Province for Cytobiology and Molecular Biotechnology, Hunan University of Chinese Medicine, Changsha, China

**Keywords:** astragali radix, angelicae sinensis radix, hemopoiesis, hematopoietic stem sell, cyclin

## Abstract

Although the compatibility of Astragali Radix (AR) and Angelicae Sinensis Radix (ASR) has favorable effect on promoting hematopoiesis in traditional Chinese medicine (TCM), the main active components and pharmacological mechanism are unknown. We investigated the five active components and its mechanisms *in vitro* and *in vivo*. Five active components of Astragalus glycosides (AST), Formononetin (FRM), Ferulic acid (FRA), Calycosin (CAL), and Calycosin-7-glucoside (CLG), which could be absorbed in intestinal tract, were detected in this study. The peripheral blood, hematopoietic growth factors (HGFs), and hematopoietic progenitor cells (HPCs) colony were observed to evaluate the effect of these five active components promoting hematopoiesis. Furthermore, hematopoietic stem cell (HSC) proliferation, aging, cycle, and related proteins were detected to explore the mechanism of these five components promoting HSC proliferation. **i)** The *in vivo* experiments showed that the combination of the five active components could remarkably increase the number of RBCs, WBCs, PLTs, and content of Hb in peripheral blood and the area of bone marrow hematopoietic tissue, as well as thrombopoietin (TPO), erythropoietin (EPO), granulocyte-macrophage colony stimulating factor (GM-CSF), and colony of CFU-GM, CFU-MK, CFU-E, and BFU-E in serum. Each of these five components promoted the recovery of RBCs and Hb, and increased TPO, CFU-MK, and CFU-E. All components except for AST increased the CFU-GM. FRA increased the number of WBCs, the area of bone marrow hematopoietic tissue, and BFU-E. FRA and AST promoted PLT recovery. FRA and CAL improved the content of GM-CSF. FRA, CAL, and CLG improved the content of EPO. **ii)** The *in vitro* experiments showed that FRA, FRM, and AST significantly promoted cell proliferation, reduced the positive rate and G0/G1 cells, and increased G2/M + S cells and the expression of cyclin D1 and CDK4 proteins in aging HSCs. Furthermore, the combination of five components had the best effect. Taken together, the five active components of AST, FRM, FRA, CAL, and CLG were the main pharmacodynamic substances of the AR-ASR compatibility, which promoted hematopoiesis. The combination of them had a synergistic effect. The mechanism of promoting hematopoiesis may be relevant to regulating cyclin-related proteins, promoting cell cycle transformation, and promoting HSC proliferation.

RETRACTED

## Introduction

The compatibility of AR with ASR is commonly used to cure disease in traditional Chinese medicine. Danggui Buxue Tang (DBT), founded in 1247 AD, is the most famous formulation and is composed of herbaceous AR and ASR in a ratio of 5:1. DBT has many pharmacological effects, such as promoting hematopoietic function (Yang et al., 2014), playing an estrogen-like effect (Xie et al., 2012), and so on. Furthermore, DBT can promote erythropoiesis, and its main active components include astragalus saponin III, AST, CAL, FRM, and FRA (Zhang et al., 2012). DBT can also promote the recovery of peripheral hemogram and bone marrow nucleated cells (BMNCs), promote the proliferation of bone marrow HPCs, and regulate the expression of HGFs, including TPO, EPO, and GM-CSF (Yan et al., 2014). Our research shows that the compatibility of AR and ASR (at ratios of 5:1, 2.5:1, 1:1, 1:2.5, 1:5, and 1:10) could increase the number of peripheral blood cells and BMNCs, enhance the content of serum HGFs and bone marrow hematopoietic tissue area, and reduce the spleen index. In particular, the compatibility of AR and ASR (ratios of 1:1, 1:2.5, and 1:5) plays the strongest role in promoting hematopoiesis. A study of an aging model of HSCs induced by tert-butyl hydroperoxide (t-BHP) discovered that AR, ASR, and their compatibility could inhibit the aging of HSCs and promote HSC proliferation and cell cycle transformation. In particular, the compatibility of AR and ASR (1:1) had the strongest effect (Zhang et al., 2017) and could promote active components [FRA, FRM, AST, CAL, and CLG (calycosin-7-glucoside)] dissolution and absorption in isolated small intestine in rats (Li et al., 2017). It is suggested that the active components (FRA, FRM, AST, CAL, and CLG) may be the main effective substances of the compatibility of AR and ASR that promote hematopoiesis. But what pharmacological effect do these active components have on hematopoiesis, respectively? Does the combination of active components have the same effect as AR and ASR on promoting hematopoiesis? And what is the mechanism promoting hematopoiesis in these active components? The answers to these questions are unclear. Therefore, in order to reveal the main pharmacodynamic substances and characteristics of the compatibility of AR-ASR on hematopoiesis, first, we studied the promoting hematopoietic action of five main components and their compatibility in bone marrow hematopoietic inhibition mice. Second, the low hematopoietic function caused by aging and chemotherapy drugs is mainly due to the reduced proliferation activity of aging HSCs. Therefore, based on the compatibility of five main active components of AR-ASR promoting hematopoietic effect, the aging model of HSCs was further adopted to study the effect of five components and their compatibility on promoting the proliferation of aging HSCs.

RETRACTED

## Materials and Methods

### Preparation of Aqueous Extract from AR and ASR

AR [*Astragalus membranaceus* BUNGE var. *mongholicus* (BUNGE), P. K. HSIAO, derived from inner Mongolia] and ASR [*Angelica sinensis* (Oliv.) Diels, Umbelliferae, originating from Gansu] (**Table 1**) were provided by the Pharmacy Department of the First Affiliated Hospital of Hunan University of Traditional Chinese Medicine and identified by Professor Zuo Yajie. Reference substances of FRA (Lot No. rq0838), FRM (Lot No. 16031005), AST (Lot No. 16022804), CAL (Lot No. 16031110), and CLG (Lot No. 16031205) were purchased from Shanghai Yuanye Biotechnology Co., Ltd. The purity of each reference substance was greater than or equal to 98%.

**Table 1:** Botanical documentation of AR and ASR.

Chinese name	Latin name	Family	Voucher number	Part used	Herbaria
Huang qi	*Astragali Radix*	*Astragalus membranaceus* Bunge var.*mongholicus* (Bge.) P.K. Hsiao	154283	Root	National Specimen Information Infrastructure (CHINA)
Dang gui	*Angelicae Sinensis Radix*	*Angelica sinensis*(Oliv.) Diels	00077426	Root	National Specimen Information Infrastructure (CHINA)

High-performance liquid chromatography was used to detect the contents of AST in AR and FRA in ASR in accordance with the description of the China pharmacopoeia, 2015 edition: the AST was more than 0.040%, and the FRA was more than 0.05%. As described in our previous method (Li et al., 2017), AR and ASR were weighted 40 g, respectively, and then placed into the circular extractor. Extract was obtained using the water reflux method after cutting. First, eight times water was added and boiled for 2 h; then, the aqueous extract was obtained after being cooled. Second, six times water was applied to the extract, boiled for 1 h, and extracted. Third, the second step was repeated. Afterward, all extracts were mixed together, filtered, and condensed with a 60°C vacuum, and the final concentration of the extract was 0.24 g/ml. Following 0.1% of sodium benzoate addition, the concentrate was sub-packaged and stored at −4°C.

RETRACTED

### Determination of Five Active Components From Aqueous Extract Using UPLC-MS

Aqueous extract (10 ml) was put into a 60°C incubator, and dry extract was created. Next, 5 ml of 70% methanol was added, and the mixture was stewed overnight after repeated shocking and mixing. The next day, the extract was shaken and mixed again, then centrifuged at 4,000 rpm for 15 min. Thereafter, the double-concentration sample consisted of the supernatant filtered by 0.22-μM Millipore filtration.

Reference substances of FRA 1.82 mg, FRM 1.83 mg, AST 2.16 mg, CAL 1.83 mg, and CLG 2.51 mg were weighed precisely and placed in a 10-ml volumetric flask and dissolved with 10 ml methanol, respectively. All reference substances were purchased from Shanghai Yuanye Biotechnology Co., Ltd. The purity of each reference substance was greater than or equal to 98%. The aqueous extract was determined by using waters-Xevo-G2-S QT of ultra performance liquid chromatography–tandem mass spectrometry (UPLC-MS) according to the manufacturer’s instructions (Acquity system, V4.1 Masslynx chromatography workstation, Waters Co., Ltd, USA).

Chromatographic conditions: ACQUITY UPLC BEH C18 chromatographic column (2.1 × 50 mm, 1.7 μm). The mobile phase: 0.1% methane acid (A); acetonitrile (B); gradient elution (0–1 min, 95→90% A; 1–4 min, 90→80% A; 4–7 min, 80→65% A; 7–10 min, 65→50% A; 10–11 min, 50→5% A; 11–12 min, 5→5% A; 12–13 min, 5→95% A; 13–15 min, 95→95% A). The column temperature was 35°C, the flow rate was 0.4 ml/min, and the injection volume was 1 μl. Based on the above conditions, UPLC fingerprints of AR and ASR aqueous extract, the reference substances of FRA, FRM, AST, CAL, and CLG, could be detected. Mass spectrometry conditions: Data were collected in the positive mode on the waters-Xevo-G2-S QT using the electrospray ionization source (ESI) (G1969-85000) in full scan mode (m/z 100–1,700). The temperature and flow rate of desolvation gas (nitrogen) were set to 325°C and 6.8 L/min, respectively. The sheath temperature and capillary voltages were 350°C and 4V, respectively.

UPLC maps of the samples and reference substances were obtained from the conditions, and the chemical structures of the five components are shown in **Figure 3**. The content of five active components from the aqueous extract was calculated by comparing the peak area between the sample and reference substance, respectively.

### Animal Models and Administration

Kunming mice (4–8 weeks old, 20–25 g, SPF class), half of which were male and half female, were provided by the Experimental Animal Center of Hunan University of Chinese Medicine, and maintained in our animal facility under controlled temperature (22–24°C) and humidity (50–60%) conditions and a 12 h light/dark cycle with free access to food and water. This study was carried out in accordance with the recommendations of the ethical standards of Guide for the Care and Use of Laboratory Animals (NRC Publications, 1996), and the protocol was approved by the Animal Ethics Committee of Hunan University of Chinese Medicine (approval no. 43004700005819, date: April 25, 2014). Animals were randomly divided into nine groups: A (blank, BLK), B (model, MDL), C (FRA), D (AST), E (FRM), F (CAL), G (CLG), H (active components combination, ACC), and I (ASR + AR, AA). Twelve mice were included in each group. The bone marrow hematopoietic function inhibition model induced by cyclophosphamide (CTX; Hengrui Medicine Co., Ltd., Jiangsu province, China; No. 16071925) was used (Li et al., 2017).

RETRACTED

All animals were fed in a clean laboratory for 2 days and administered as follows. The mice in the blank group were given sodium carboxymethylcellulose (25 ml/kg) intragastrically each day for 7 days. The model group was gavaged as above while receiving an intraperitoneal injection of CTX (360 mg/kg) on the third day for 3 days, and materials were taken on the eighth day. All drug groups were treated with drug for 7 days from the first day and received the CTX injection on the third day. All animals were anaesthetized with isoflurane and then sacrificed, and materials were taken at 24 h after the last administration.

The administered dosage of the five active components was determined by referring to the content of the five active components in the AR-ASR (ratio of 1:1) aqueous extract. The dosage of each active component was the same as that of the five active components in the aqueous extract with simple or combined use. As our previous experiments (Li et al., 2017), the gavaged dose of crude drugs was 6 g/kg in mice. According to the content of the five main active components in aqueous extract (**Table 2**), the dosage of the five active components was as follows: FRA 574.74 μg/kg, FRM 607.26 μg/kg, AST 275.52 μg/kg, CAL 391.26 μg/kg, and CLG 1394.28 μg/kg. The dose of active components combination was the same as that of each active component using along. The set point of gavaged capacity was 25 ml/kg in mice, so the concentrations of the five active components in the mixture were as follows: FRA 23 μg/ml, FRM 24 μg/ml, AST 11 μg/ml, CAL 16 μg/ml, and CLG 56 μg/ml. Each standard substance was accurately weighed and then blended with 0.4% sodium carboxymethylcellulose for use.

**Table 2:** Content of five active components in AR and ASR aqueous extract.

Active Component	Peak Area of Sample	Peak Area of Reference Substance	Concentration in Reference Substance (mg/ml)	Content in Extract (µg/ml)	Content in Crude Drug (µg/g)
**FRA**	4139081.13	16383292.89	0.182	22.99	95.79
**FRM**	21478556.5	178291095.4	0.216	24.29	101.21
**AST**	858379.75	3815896.35	0.183	11.02	45.92
**CAL**	19993881.08	116689546.3	0.183	15.68	65.33
**CLG**	15800322.32	35555498.02	0.251	55.77	232.38

RETRACTED

### Peripheral Blood Assay

At 24 h after the last administration, 500 μl of blood by heart puncture was put into a test tube containing ethylenediaminetetraacetic acid (EDTA; Lot No. WB07014, Well Biological Science Co., Ltd, Hunan Province, China), and the numbers of red blood cells (RBCs), white blood cells (WBCs), and platelets (PLTs) as well as the hemoglobin (Hb) content were detected by automatic blood cell analyzer (UniCel^®^ DxH 800 Coulter, Beckman Coulter, Co., Ltd., USA).

### Determination of Serum HGF Using ELISA Kits

Five hundred microliters of blood by heart puncture was put into sterile tubes after coagulation and then centrifuged at 3,000 rpm for 10 min at 4°C. The upper serum was obtained and stored at –80°C. Afterward, the contents of EPO (Cloud-Clone Corp, Lot No. L161124009), TPO (Cloud-Clone Corp, Lot No. L161130210), and GM-CSF (ExCell Bio, Lot No. 21S343) were detected using enzyme-linked immunosorbent assay (ELISA) kits (Cloud-Clone Corp, Lot No. L161124009).

### Detection of Bone Marrow Hematopoietic Tissue Area

The femur was isolated from the left hind leg at 24 h after the last administration and then fixed in 10% neutral formaldehyde for 3 days, washed for 45 min, and subsequently decalcified in EDTA for 40 days. Afterward, the femur was gradient dehydrated using ethanol after washing, made transparent using xylene, paraffin embedded, then cut into 5-μm slices from the 2-mm position under the caput femoris. Next, the slices were affixed to a slide treated with polylysine, dyed with hematoxylin and eosin (H&E) staining after dewaxing, gradient dehydrated using ethanol, and made transparent using xylene; the slide was sealed with neutral resins. Afterward, the percentage of the bone marrow hematopoietic tissue area of the bone marrow cavity was calculated using Image-Pro Plus software.

### HPC Culture and Count

At 24 h after the last administration, the right hind leg of the mice was obtained and soaked in 75% alcohol and washed with phosphate-buffered saline (PBS; Genom, Lot No. GNM20012). Afterward, the muscles and connective tissue were removed, and the femur was separated. Then, the femur was removed to collect the bone marrow, and the cells in the marrow cavity were rushed out with 3 ml of IMEM (Gibco, Lot No.1846253) and repeatedly blown out and dispersed. They were then centrifuged 3,000 rpm for 8 min at 4°C, and the supernatant was removed. Subsequently, 2 ml of IMEM was added, which was blown and mixed repeatedly, and 10 μl of cell solution was diluted 10 times and counted after being screened with a 200 mesh cell strainer. The concentration of cells in each group was adjusted to 2 × 10^5^/ml. According to our previous method (Li et al., 2017), the prepared BMNCs were fully mixed with the culture system and added to the six-well cell culture plate, then cultured at 37°C, 5% CO_2_, and saturated humidity. Each well contained 1 ml of culture solution (**Table 3**). The erythrocyte–colony-forming unit (CFU-E) was observed and counted on the third day of culture. Burst forming unit–erythrocyte (BFU-E), granulocyte-macrophage colony-forming unit (CFU-GM), and megakaryocyte colony-forming unit (CFU-MK) were observed and counted on the seventh day. BFU-E and CFU-E were identified by 2-methoxy benzidine staining as red positive cells. For BFU-E, > 50 cells and, for CFU-E, > 8 cells were identified as a colony. CFU-GM was dyed red with NAS-DCE as a positive cell, and greater than 50 cells were considered a colony. CFU-MK was stained by acetylcholinesterase and identified as a colony if the cell was brown, and there were greater than three cells (**Figure 1**). The colony number was calculated as the total colonies in every well.

RETRACTED

**Table 3:** Constituents of the CFU-GM, CFU-MK, CFU-E, and BFU-E culture systems.

Constituent	CFU-GM	CFU-MK	CFU-E	BFU-E
β-mercaptoethanol (10^–3^ M, ml)	0.01	0.01	0.1	0.1
3% L-glutamine (ml)	0.015	0.015	0.015	0.015
Horse sera (ml)	0.25	0.4	0.25	0.25
rhGM-CSF (50 ng/ml, ml)	0.15	—	—	—
rhEPO (20 U/ml, ml)	—	0.05	0.05	0.1
IL-3 (20 ng/ml, ml)	—	0.05	—	0.05
mTPO (5 ng/ml, ml)	—	0.1	—	0.1
Bone marrow nucleated cell	1 × 10^5^	1 × 10^5^	1 × 10^5^	1 × 10^5^
IMDM media (ml)	To 0.9	To 0.9	To 0.9	To 0.9
3% Agar (ml)	0.1	0.1	0.1	0.1

**Figure 1:** Staining identification of progenitor cells (magnification: X 400) **(A)** BFU-E, red cells were positive cells; **(B)** CFU-GM, bright red cells were positive cells; **(C)** CFU-E, red cells were positive cells; **(D)** CFU-MK, brown cells were positive cells. Scale bars, 50 µm.

### Preparation of Drug-Containing Plasma

The drug-containing plasma was prepared according to that described in the literature (Chen et al., 2011). Male adult Sprague-Dawley rats (8 weeks old; 180–200 g, SPF class) were provided by the Experimental Animal Center of Hunan University of Chinese Medicine and fed as previously mentioned. Rats were randomly divided into blank control and drug groups, each consisting of 10 rats. The rats of the blank control were fed with distilled water, and the rats of the other groups were fed with ASR-AR 38 g/kg (AR: ASR = 1:1). All rats were administered at 9 am and 4 pm, respectively, each day. After seven consecutive gavages, these rats were anaesthetized with isoflurane and blood was drawn from a common carotid artery 2 h after the last medicine administration and anticoagulated with 2% EDTA-Na_2_ (blood: anticoagulant = 9:1). The blood was then centrifuged at 4°C at 3000 rpm for 15 min. The plasma in the same group was equally blended, filtrated, and stored at −80°C.

RETRACTED

### BMNC Culture and Sorting

The femur and tibia were isolated under sterile conditions after the mice were sacrificed. Single-cell suspension was obtained after repeatedly rinsing the marrow cavity with PBS (containing 2 mmol/L EDTA, 0.5% bovine serum, albumin, pH 7.4), then added to the top of the lymphocyte separation solution, and centrifuged at 2,000 rpm for 20 min. The middle white layer was then drained into the new centrifugal tube after three washes with PBS, and the BMNCs were on standby. Afterward, the BMNCs were added into 90 μl of PBS and 10 μl of anti-Sca-1-PE (Miltenyi, Lot No. 130102297) and incubated at 4°C for 10 min, and then supernatant was abandoned after centrifugation at 800 rpm for 5 min, added to 80 μl of PBS and 20 μl of anti-PE Micro Beads (Miltenyi, Lot No. 130048701), and finally incubated at 4°C for 10 min. To abandon the supernatant after centrifugation at 800 rpm for 5 min again, the BMNCs were resuspended with 0.5 mL of PBS and injected into magnetic separation column (Miltenyi, Lot No. 130042201). The unlabeled cells collected in the outflow tract were sca-1^-^ cells after three washes with PBS, and the sca-1^+^ cells stayed in the column. The labeled cells washed out with 0.5 ml of PBS from the separation column were sca-1^+^ HSCs. A total of 1 × 10^6^ of HSCs labeled with anti-sca-1-PE before and after sorting were collected, and the positive rate of sca-1^+^ HSCs was detected by flow cytometry. Results showed that the positive rate of sca-1^+^ HSCs before sorting was 3.6%, and the positive rate was 92.39% after sorting (**Figure 2**), which suggested that the purity of the sca-1^+^ HSCs increased significantly after magnetic bead sorting.

**Figure 2:** The positive rate of sca-1+ HSCs was detected by flow cytometry. **(A)** Percentage of sca-1+ HSCs before sorting in 3.6% **(B)** Percentage of sca-1+ HSCs after sorting is 92.39%.

### HSC Culture and Generation

The HSCs (more than 90% positive rate) were resuspended with 10 mL IMDM (containing 10% fetal bovine serum, 100 UL/L penicillin, 100 g/l streptomycin) after PBS washes. The cell density was adjusted to 2 × 10^5^/ml and inoculated in a culture flask at 4°C in 5% CO_2_, 95% O_2_ atmosphere. As the color of the culture solution was dodged, the culture solution was centrifuged at 800 rpm for 5 min, and then supernatant was abandoned and cultured with new solution at 37°C in a 5% CO_2_, 95% O_2_ atmosphere. The cell culture solution in the flask was placed into the tube and centrifuged at 800 rpm for 5 min, then the supernatant was abandoned, and cells were counted after resuspending with solution. The cell density was adjusted to 2 × 10^5^/ml and inoculated in a culture flask at 4°C in a 5% CO_2_, 95% O_2_ atmosphere. The cells were passaged four to six generations for the experiment.

RETRACTED

### CCK-8 and SA-β-Gal Assay

HSCs of four to six generations were inoculated into 96-well plates and synchronized G0 phase cultured with serum-free culture medium for 12 h, then senescence was induced with t-BHP (100 μmol/L) culture medium and treated with active components in different concentrations for 24 h. The active components of the cell cultures were prepared as follows: FRM, AST, CAL, and CLG were dissolved into a reserve solution with 0.1% dimethyl sulfoxide (DMSO)–PBS (Lot No. ST038, Sigma, USA), and FRA was dissolved into reserve solution with 0.1% DMSO-IMDM (Lot No. 12440046, Hyclone, USA), for dilution with cell culture medium as required, and the final concentration of DMSO in the medium was 0.1%. The proliferative activity of HSCs was detected by assaying the optical density (OD) value of a 450-nm laser using cell counting kit-8 (CCK-8; Boster, Lot No. AR1160-500). The rate of HSC proliferation was calculated by the following equation: proliferation rate (%) = [(OD of drug-treated − OD of CTL) − 1] × 100%.

After determining the effect of active components on HSC proliferation, three components (FAR, AST, and FRM) were chosen as the basic factor. We observed the influence of the basic factor and CAL and CLG on HSCs using the L4(2^3^) orthogonal experiment and analyzed the synergism of each component on HSCs (**Tables 4**, **5**). HSCs of four to six generations were inoculated into 96-well plates, and the cells were synchronized G0 phase cultured with serum-free culture medium for 12 h and then cultured with complete medium containing t-BHP for 24 h. CCK-8 was then used to assay the cell proliferation rate, and the SA-β-Galactosidase Staining Kit (Beyotime, Lot No. C0602) was used to detect cell senescence. Four hundred cells were counted, and the positive cells appeared blue under the inverted microscope; the negative cells had no color. The rate of positive cells (%) = (the number of positive cells/the number of total cells) × 100%. The rate of positive cells was the aging rate.

RETRACTED

**Table 4:** Factors and levels of orthogonal experiments.

Levels	Factors		
	Basal factors (BF)	CAL	CLG
1	Use	Use	Use
2	Use	Not	Not

There are three factors (BF, CAL, CLG) and two levels: the basal factors include FRA, FRM, and AST, and the levels are divided into two situations: use or not.

**Table 5:** Orthogonal test results and analysis.

No.	1 (CAL)	2 (CLG)	3 (CAL × CLG)	Drug Constituents	Proliferation Rate (%)	Aging Rate (%)
1	1	1	1	BF+CAL+CLG	86.16 ± 4.67••^##^	22.87 ± 1.69••^##^
2	1	2	2	BF+CAL	63.46 ± 3.06•**^##^	43.08 ± 2.56••*^##^
3	2	1	2	BF+CLG	61.06 ± 1.67•*^##^	45.64 ± 4.62•**^##^
4	2	2	1	BF	47.13 ± 3.90**^##^	53.57 ± 3.21**^##^
5	/	/	/	/	0.00 ± 0.00^∆∆^	78.61 ± 6.43^∆∆^
6	/	/	/	/	52.54 ± 2.33	5.04 ± 3.21
Σ1	149.62	147.22	86.16	/	/	/
Σ2	108.19	110.59	171.65	/	/	/
R	41.43^★^	36.63^★★^	85.49^★★^	/	/	/
Σ′1	65.95	68.51	21.87	/	/	/
Σ′2	99.21	96.65	142.29	/	/	/
R′	33.26^★^	28.14^★★^	120.42^★★^	/	/	/

There were four combinations in the L_4_(2^3^) orthogonal design, so drugs were constituted as follows: No. 1 was treated with BF+CAL+CLG, No. 2 was treated with BF+CAL, No. 3 was treated with BF+CLG, No. 4 was treated with BF. In addition, No. 5 and No. 6 were not treated with drugs. No. 1-5 used t-BHP–induced cells, No. 6 used normal cells. The proliferation rate assay was similar to that in **Figure 8**. SA-β-Galactosidase Staining Kit was used to detect cell senescence; 400 cells were counted, and the positive cells appeared blue under the inverted microscope, whereas the negative cells had no color. The rate of positive cells (%) = (the number of positive cells/the number of total cells) × 100%. The rate of positive cells equaled the aging rate. Σ1, the proliferation rate sum of level-1 effect; Σ2, the proliferation rate sum of level-2 effect; R, the range of proliferation rate; Σ′1, the aging rate sum of level-1 effect; Σ′2, the aging rate sum of level-2 effect; R′, the range of proliferation rate. The data are presented as the mean ± SD. N = 4. ^∆∆^P < 0.01 vs. CTL, ^##^P < 0.01 vs. model, *P < 0.05, **P < 0.01 vs. BF. •P < 0.05, ••P < 0.01 vs. BF+CAL+CLG, ^★^P < 0.05, ^★★^P < 0.01 level-1 vs. level-2 among three factors.

After determining the active components’ combination in HSC proliferation, we designed 10 groups: A, control group (CTL); B, model group (MDL); C, blank plasma group (BP; 10% concentration); D, FRA group (9 μg/ml); E, AST group (8 μg/ml); F, FRM group (6 μg/ml); G, CAL group (10 μg/ml); H, CLG group (10 μg/ml); I, active components combination group (ACC: FAR 9 μg/ml + AST 8 μg/ml + FRM 6 μg/ml + CAL 10 μg/ml + CLG 10 μg/ml); and J, drug containing plasma group (DCP; 10% concentration). HSCs of four to six generations were inoculated into 96-well plates and synchronized G0 phase cultured with serum-free culture medium for 12 h and then cultured with complete medium containing t-BHP for 24 h. Meanwhile, we joined the different active components or drug-containing plasma into medium: groups A, B, and C joined blank plasma; groups D, E, F, G, H, and I joined different efficient composition; group J joined the drug containing plasma. Afterward, we assayed the proliferation rate with CCK-8 as previously mentioned, and SA-β-Gal was used to detect cell senescence.

RETRACTED

### Flow Cytometry Assay

Flow cytometry was used to detect the cell cycle distribution in each group. A total of 1 × 10^6^ of HSCs were collected after centrifugation, washed once with 1 ml PBS, fixed with 70% ice ethanol overnight, and incubated at 37°C for 30 min with 100 μl bovine pancreas DNasel (Bp DNasel, 1 g/l). Afterward, cells were stained with 1 ml propidium iodide (final concentration 50 μg/ml prepared with 0.01 mol/L PBS) away from light at 4°C for 30 min, and the cell number was not less than 2 × 10^5^. The percentage of cells (G0 phase, G1 phase, G2 phase, S phase, M phase) were counted; the cells at the G0 and G1 phase were quiescent cells, and the cells at the G2, S, and M phases were proliferating phase cells.

### Western Blot Analysis

Cells were collected after centrifugation and abandoning supernatant and then washed twice with PBS, and cell pellet was collected again. Next, the RIPA lysate was added, and ice cracked for 10 min after blending, then supernatant was collected after centrifugation at 12,000 rpm at 4°C for 30 min. The concentration of protein was assayed by bicinchoninic acid protein assay kit. First, the concentration of each sample protein was adjusted to 2 μg/μl, and then sodium dodecyl sulfate–polyacrylamide gel electrophoresis loading buffer was added 5 times, bathed in boiling water for 5 min, and cooled down for use. Second, to prepare the separation and stacking gels, 20 μl of the sample was joined into the sample hole. Electrophoresis separation was implemented and wetly transferred to polyvinylidene fluoride nitrocellulose membrane. Blocking was then performed with 5% tris-buffered saline (TBS) and Tween 20 (TBST) buffer. The membrane was then incubated with cyclin dependent kinase 4 (CDK4) antibody (ab199728, 1:2,000, Abcam), cyclin D1 antibody (No. 04-1151, 1:10,000 Abcam), and β-actin antibody (No. 60008-1-Ig, 1:5,000, Abcam) at 4°C overnight. Afterward, the membrane was washed with TBST three times for 10 min each time, followed by incubation with goat anti-rabbit horseradish peroxidase horseradish peroxidase (HRP)-labeled IgG (ab205718, 1:6,000, Abcam, used for measurement of CDK4 and cyclin D1) or rabbit anti-rat HRP-labeled IgG (ab205719, 1:5,000, Abcam, used for measurement of β-actin) at room temperature for 2 h. The membrane was washed with TBST three times for 10 min each time, with enhanced chemiluminescence Western blotting detection in response. The X-ray film was placed into the image analysis system of the Gel Doc2000 to determine the integral OD (IOD) of the objective band, taking β-actin as an internal reference and taking the ratio of the IOD values of the protein objective band and the β-actin protein objective band as the relative expression of target protein.

RETRACTED

### Statistical Analysis

Statistical package SPSS 17.0 (SPSS Inc., Chicago, IL, USA) was used for all analyses. Data were expressed as mean ± standard deviation. One-way analysis of variance was used for multigroup comparisons, and the least significant difference test or Dounnett’s T3 test was used for two-group comparison. The L4(2^3^) orthogonal test adopted the variance analysis of the orthogonal test to determine the interaction between the basic factors and minor factors. Values of *p* < 0.05 were considered statistically significant.

## Results

### Determination of Five Active Components of Aqueous Extract

The contents of the five main active components were measured by UPLC-MS. The contents of the five main active components were calculated by comparing the peak area of each component to reference substances. Results showed that the five active components had the same chromatogram no matter the aqueous extract (**Figure 3I**) or reference substance (**Figure 3II**). The contents of the five active components in the aqueous extract are shown in **Table 1**.

**Figure 3:** UPLC-MS assay of the 5 main active components. **(I)** UPLC fingerprints of the five components in each reference substance (left). The peak time was evaluated using UPLC assay, and peak of each component is indicated by an arrow **(A)** The peak time of FRA was 12 min, **(B)** The peak time of FRM was 21 min, **(C)** The peak time of AST was 21 min, **(D)** The peak time of CAL was 17 min, **(E)** The peak time of FRA was CLG 11 min. **(II)** UPLC fingerprints of five components of aqueous extract (right). The peak time was evaluated using UPLC assay, and peak of each component is indicated by an arrow. **(A)** The peak time of FRA was 12 min, **(B)** The peak time of FRM was 21 min, **(C)** The peak time of AST was 22 min, **(D)** The peak time CAL was 17 min, **(E)** The peak time of FRA was CLG 11 min. a, FRA; b, FRM; c, AST; d, CAL; e, CLG.

RETRACTED

### ACC Improves Peripheral Hemogram and Increases the Area of Bone Marrow Hematopoietic Tissue

We used a mouse model of bone marrow hematopoiesis suppression induced by CTX (Li et al., 2017). In comparison with the BLK group, blood assay showed a significant decrease in WBC, PLT, RBC, and Hb (**Figures 4a-d**), and the area of bone marrow hematopoietic tissue diminished in the model group (**Figures 4e, f**).

**Figure 4:** ACC improved the peripheral hemogram and added the area of bone marrow hematopoietic tissue. **(a–d)** A total of 500 uL of blood by heart puncture was put into the tube contatining EDTA, RBC, WBC, PLT, and Hb were measured with an automated hematology analyzer, respectively. **(e)** Bone marrow hematopoietic tissue was observed with a microscope, and the percentage of hematopoietic tissue area to marrow cavity was compared with Image-Pro Plus. The data are presented as mean ± SD. N = 12. ^∇∇^ *P* < 0.01 vs BLK, ^#^ *P* < 0.5, ^##^ *P* < 0.01 vs. MDL, *P <0.05, **P < 0.01 vs. ACC. **(f)** The area of bone marrow hematopoietic tissue in each group (H&E staining, magnification: 100 X). Three visual fields were obtained in each slide by microscope. The percentage of the bone marrow hematopoietic tissue area in the bone marrow cavity area was calculated using Image-Pro Plus software and the mean value as the bone marrow hematopoietic tissue area. The data are presented as the means ± SD. N = 12. Scale bards, 500 µm. A, CTL; B, MDL; C, FRA;D, AST; E, FROM; F, CAL; G, CLG; H, ACC; I, AA.

To reveal whether ACC has a protective role against CTX-induced hematopoiesis suppression, we applied the active components (exclusive or compatibility use) to model mice for 8 days. Blood assay showed that WBCs were significantly increased in the FRA, ACC, and AA groups compared with the model. In comparison with the ACC group, WBCs were significantly decreased in the FRM, CAL, and CLG groups, but there was no difference in AST, ACC, and AA groups (**Figure 4a**).

PLTs were significantly increased in the AST, FRA, ACC, and AA groups compared with the model. In comparison with the ACC group, PLTs were significantly decreased in the FRM and CLG groups, but there was no difference in the AST, CAL, ACC, and AA groups (**Figure 4b**).

The RBCs and Hb were significantly increased in the AST, FRA, FRM, CAL, CLG, ACC, and AA groups compared with the model group. In comparison with the ACC group, there was no difference in any of the drug groups (**Figures 4c, d**).

Image-Pro Plus analysis showed that compared with the model, the area of bone marrow hematopoietic tissue was enlarged in the FRA, ACC, and AA groups. In comparison with the ACC group, the area of bone marrow hematopoietic tissue was significantly decreased in the AST, FRA, FRM, CAL, and CLG group, but there was no difference in the AA group (**Figures 4e, f**). These data suggest that ACC could improve the inhibition of hematopoiesis function by adjusting the peripheral hemogram and increasing the area of bone marrow hematopoietic tissue, and the effect of ACC and AA was equal.

RETRACTED

### ACC Increases the Level of HGFs in Serum

HGFs (including EPO, TPO, and CSF), a series of cytokines acting directly on bone marrow HPCs, could promote HPC proliferation, directional differentiation, and maturation. In addition, HGFs could affect many aspects of the hematopoiesis process, thus regulating the survival, growth, and development of primitive blood cells.

As compared with controls, the levels of EPO, TPO, and CSF were remarkably decreased in CTX-treated mice (**Figures 5A–C**). We explored the effect of all drugs on HGFs, and the results showed that compared with the model, the GM-CSF level was remarkably increased in some drug-treated groups (FRA, CAL, ACC, and AA; **Figure 5A**), the EPO level was dramatically increased in some drug-treated groups (FRA, CAL, CLG, ACC, and AA; **Figure 5B**), and the TPO level was dramatically increased in all drug-treated groups (**Figure 5C**). As compared with the ACC group, the levels of EPO (AST, FRM group), TPO (AST, FRM group), and GM-CSF (FRA, AST, FRM, CLG group) were decreased in serum, yet there was no difference in the other groups. These results indicate that the ACC could promote HPC proliferation by increasing the level of HGFs, and the effect of ACC and AA was equal.

**Figure 5:** ACC increases the level of HGFs in serum. **(A)** Content of GM-CSF in the serum in each group. **(B)** Content of TPO in serum in each group. **(C)** Content of EPO in serum in each group. The data are presented as mean ± SD.N = 12. ^∇^ *P* < 0.05 vs. CTL; ^∇∇^ *P* < 0.01 vs. CTL, ^#^ *P* < 0.05, ^##^ *P* < 0.01 vs. MDL, *P < 0.05, **P < 0.01 vs. ACC. A, CTL; B, MDL; C, FRA; D.AST, E. FMlF, CAL; G, CLG; H, ACC; I, AA.

### ACC Increases HPC Colony

Results showed that compared with CTL, the CFU-GM, CFU-MK, CFU-E, and BFU-E were all significantly decreased in the CTX-treated model (**Figures 6A–D**). The CFU-GM was significantly increased by ACC and other drug (FRA, FRM, CAL, CLG, AA) intervention in comparison with the model and was decreased in other drug groups (AST, FRM) in comparison with the ACC group. However, there was no difference among the FRA, CAL, CLG, AA, and ACC groups (**Figure 6A**). CFU-MK was significantly increased by ACC and other drug (FRA, FRM, CAL, CLG, AA) intervention in comparison with the model; however, there was no difference among the CAL, AA, and ACC groups (**Figure 6B**). The CFU-E was significantly increased by ACC and other drug (FRA, AST, FRM, CAL, CLG, AA) intervention in comparison with the model. Compared with the ACC group, the CFU-E was remarkably decreased in other drug groups (AST, FRM, CAL, CLG); however, there was no difference between the FRA and AA groups (**Figure 6C**). Similarly, the BFU-E was significantly increased by ACC and other drug (FRA, AA) interventions in comparison with the model and decreased in other drug groups (AST, FRM, CAL, CLG) in comparison with the ACC group. However, there was no difference among the FRA, AA, and ACC groups (**Figure 6D**). These results imply that ACC could promote HPC colony proliferation, and the effect of ACC and AA was equal.

RETRACTED

**Figure 6:** ACC increases hematopoietic progenitor cells colony. **(A–B)** The mice were gavaged with saline (25 ml/kg) in the control group (CTL) and model group (MDL) for 7days. **(C–I)** The mice were gavaged with drugs, respectively, for 7 days. To count the number of colonies under the microscope, we countedmore than eight cells as a colony in CFU-E, more than 50 cells as a colony in BFU-E and CFU-GM, more than three cells as a colony in CFU-MK, and the colony number of HPCs is the total colonies of every well under microscopes. **(A)** The comparison of CFU-GM count under microscopes in each group. **(B)** The comparison of CFU-MK count under microscopes in each group. **(C)** The comparison of CFU-E count under microscopes in each group. **(D)** The comparison of BFU-GM count under microscopes in each group. The data are presented as mean ± SD.N = 12. ^∇^ *P*<0.05 vs. CTL; ^∇∇^ *P*<0.01 vs. CTL, ^#^ *P*<0.05, ^##^ *P*<0.01 vs. model, *P<0.05, **P<0.01 vs. ACC. A, CTL; B, MDL; C, FRA; D, AST; E, FRM; F, CAL; G, CLG; H, ACC; I, AA.

### Five Active Components Promote HSC Proliferation

To explore the effect of five active components from AR and ASR on HSCs, we use the t-BHP induced model of cell senescence according to the methods detailed in the literature (Ungvari et al., 2013). The naturally growing cells were the CTL, and the t-BHP induced cells were the MDL (the rate of proliferation was zero). In comparison with MDL, FRA, AST, and FRM could promote proliferation of aging HSCs and presented a dose–effect relationship with the increase of drug concentration (FRA concentration from 2.25 to 18 μg/ml, AST concentration from 2 to 16 μg/ml, FRM concentration from 1.5 to 12 μg/ml). However, there was no similar action in CAL (the concentration from 2.5 to 40 μg/ml) and CLG (the concentration from 1.25 to 20 μg/ml; **Figure 5**). Taken together, these results provide proof that FRA, AST, and FRM are the main effective components of AR and ASR that promote HSC proliferation (**Figure 7**).

RETRACTED

**Figure 7:** Effect of five active components on aging cell proliferation. HSCs of 4–6 generations were inoculated into 96-well plates, and the cells were synchronized G0 phase cultured with serum-free culture medium for 12 h, then treated with t-BHP(100 µmol/L) and joined different concentrations of the five active components in each drug group, respectively, for 24 h. Next, the cells’ proliferative activity was detected by assaying the OD value of a 450-nm laser using CCK-8. The rate of HSCs proliferation was calculated by the following equation: proliferation rate (%) = [(OD of drug-treated–OD of CTL)-1] x 100%. The HSCs were pretreated with t-BHP in the MDL and drug groups, and nontreated HSCs were used as CTL (**Figure A–E**). **(A)** The t-BHP-treated HSCs proliferation. **(C)** The effect of AST (0, 2, 4, 8, 16, 32 µg/ml) on t-BHP treated HSCs proliferation. **(D)** The effect of CAL (0, 2.5, 5, 10, 20, 40 µ g/mL) on t-BHP-treated HSCs proliferation. **(E)** The effect of CLG (0,1.25, 2.5, 5, 10, 20 µg/ml) on t-BHP-treated HSCs proliferation. The data are presented as the mean ± SD. N = 4.

### ACC Promote HSC Proliferation and Resist HSCs Aging

After determining the main active components of five components, we chose the effective concentration that could remarkably promote HSC proliferation. The basal factors (main components) included FAR (9 μg/ml), AST (8 μg/ml), and FRM (6 μg/ml), and the secondary factors (minor components) included CAL (A, 10 μg/ml) and CLG (B, 10 μg/ml). To search for the best combination, we adopted the L4(2^3^) orthogonal experiment (**Table 3**). The results showed that the combination of basal factors (BF) can significantly promote HSC proliferation and reduce cell senescence rate; the same effect of BF + A and BF + B was superior to the BF. Similarly, the effect of BF + A + B was significantly better than the above three combinations (**Table 4**). The interaction analysis indicated that the effect of the BF was 47.13% in the cell proliferation rate, the effect of BF + A = 63.46% − 47.13% = 16.33%, the effect of BF + B = 61.06% − 47.13% = 13.93%, the effect factor of BF + A + B = 86.16% − 41.13% = 39.03% > [(BF + A) + (BF + B)], which suggest that these five components have the synergistic effect on promoting HSC proliferation.

In cell senescence rate, the effect of the BF was 53.57%, inhibition effect on aging rate of BF + A = 53.57% − 43.08% = 10.49%, the inhibitory effect of BF + B = 53.57% − 45.64% = 7.93%, inhibition effect of BF + A + B = 53.57% − 22.87% = 30.70% > [(BF + A) + (BF + B)], which suggest that these five components have the synergistic effect on inhibiting HSC senescence.

RETRACTED

After determining the synergistic effect of the main components (FAR, AST, FRM) and minor components (CAL, CLG) on promoting HSC proliferation and restraining the HSC senescence, we designed the experiment to assay the effect of drug containing plasma on HSC proliferation and aging. Results showed that compared with MDL or BP, the rate of HSC proliferation was remarkably enhanced and the rate of HSC senescence was remarkably decreased in the drug groups (FAR, FRM, AST, ACC, DCP). The effect of ACC was stronger than in the other five active components groups (FAR, FRM, AST, CAL, CLG), and there was no difference between ACC and DCP (**Figure 8**).

**Figure 8:** **(I)** Aging HSCs induced by t-BHP were improved bt drug treatment. Aging cells were assayed by SA-β-galactose glucoside enzyme staining method. The positive cells are indicaed by blue (arrow). Magnification: 400x. Scale bars. 50 µm. **(II)** The influence of each drug on HSC aging and proliferation. After determining the effective synergistic compatibility of the main components (FAR, AST, FRM) and minor components (CAL, CLG) on HSCs proliferation, HSCs of 4-6 generations were inoculated into 96-well plates and synchronized G_0_ phase cultured with serum-free culture medium for 12 h, then cultured with complete medium containing t-BHP for 24 h. Meanwhile, we joined the different active ingredients or drug containing plasma into medium. There were 10 groups: **(A)** Blank group (BLK), **(B)** model group (MDL), **(C)** blank plasma group (BP), **(D)** FRA group (9 µg/ml), **(E)** AST group (8 µg/ml), **(F)** FRM group (6 µg/ml), **(G)** CAL group (10 µg/ml), **(H)** CLG group (10 µg/ml), **(I)** ACC group (FAR 9 µg/ml + AST 8 µg/ml + FRM 6 µg/ml + CAL 10 µg/ml + CLG 10 µg/ml), **(J)** drig containing plasma (DCP) group (AR 19 g/kg + ASR 19 g/kg). Groups A, B, and C joined the blank plasma, and groups D, E, F, G, H, and I joined different efficient compositions, respectively. Group J joined the drug containing plasma. Afterward, to assay the proliferation rate with CCK-* as previously mentioned, 400 cells was tha aging rate. The data are presented as the means ± SD. N = 4 ^∇∇^ *P*<0.01 vs. BLK, ^##^ *P* < 0.001 vs. model, *P <0.05, **P<0.001 vs. ACC, ^••^ *P*<0.01 vs. BP. A, CTL; B, MDL; C, BP; D, FRA; E, AST; F, FRM; G, CAL; H, CLG; O, ACC; J, DCP.

### The Influence of ACC on Cell Cycle of Aging HSCs Induced by t-BHP

Flow cytometry was used to detect the cell cycle distribution in each group. Compared with CTL, the cells of the G0/G1 phase remarkably increased, and the cells of the G2/M + S phase significantly decreased in MDL and BP. In comparison with MDL and BP, the cells of the G0/G1 phase remarkably decreased, and the cells of the G2/M + S phase significantly increased in FRA, FRM, AST, ACC, and BP. Compared with ACC, the cells of the G_0_/G_1_ phase remarkably increased, and the cells of the G2/M + S phase significantly decreased in FRA, FRM, AST, CAL, and CLG groups, yet there were no differences between ACC and BP (**Figure 9**).

RETRACTED

**Figure 9:** The influence of each drug on HSC cycle. Cell cycle was determined by flow cytometry, 1 x 10^6^. HSCs were collected after centrifugation, washed once with 1 ml PBS, fixed with 70% ice ethanol overnight, and incubated at 37ºC for 30 min with 100 µl bovine pancreas DNasel (Bp DNasel, 1g/l). Afterward, cells were stained with 1 ml propidium iodide (PI) away from light at 4ºC for 30 min, and the cell number was not less than 2 x 10^5^. The percentage of cells (G0 phase, G1 phase, G2 phase, S phase, M phase) was counted, respectively, and the cells at the G0, G1 phase were quiescent cells and the cells at the G2, S, and M phases were proliferating phase cells. The percentage of cells in G0, G1, G2, S and M phases was counted, and the cells in the G0/G1 phase were quiescent cells, whereas the other cells in the G2, S, and M phases were proliferating cells. The data are presented as the means ± SD.N = 4. ^∇∇^ *P*< . 01 vs. CTL, ^##^ *P* < 0.01 vs. model, *P<0.05, **P<0.01 vs. ACC, •*P*<0.05 vs. BP. A, CTL; B, MDL; C, BPl; D, FRA; E, ASTL; F, FRM; G, CAL; H, CLGL; I, ACC; J, DCP.

### The Influence of ACC on Cyclin D1 and CDK4

The protein levels of cyclin D1 and CDK4 were assessed using Western blot. Compared with CTL, cyclin D1 and CDK4 protein remarkably decreased in MDL and BP. In comparison with MDL, cyclin D1 and CDK4 protein remarkably increased in FRA, FRM, AST, and ACC groups. Compared with ACC, cyclin D1 and CDK4 protein remarkably decreased in the FRA, FRM, AST, CAL, and CLG groups. Compared with BP, cyclin D1 and CDK4 protein remarkably increased in DCP, and there were no differences between the ACC and DCP groups (**Figure 10**).

**Figure 10:** **(I)** The influence of each drug on HSC cyclin D1 and CDK4. The protein level of cyclin D1 and CDK 4 was assessed using Western blot. The integrated optical density of target bands. The data are presented as the means ± SD.N = 4 ^∇^ *P*<0.05 vs. CTL; ^∇∇^ *P*<0.01 vs, CTL, ^##^ *P*<0.01 vs. model, *P<0.05, **P<0.01 vs. SAI, ^•^ *P*<0.05 vs. BP. A, CTL; B, MDL; C, BP; D, FRA; E, AST; F, FRM; G, CAL; H, CLG; I, ACC; J, DCP. **(II)** The expression profiles of cyclin D1 and CDK 4 proteins in each group were detected by Western blot. A, CTL; B, MDL; C, BP; D. ACC; E, DCP; F, FRA; G, AST; H, FRM; I, CAL; J, CLG.

RETRACTED

## Discussion

In Chinese medicine, the combination of AR-ASR (5:1) had the strongest effect on promoting hematopoietic function as curing anemia. For example, DBT could not only inhibit the decrease in immunologically mediated blood cells but also stimulates the growth of bone marrow cells and promotes the proliferation of CFU-GM, CFU-E, and BFU-E in bone marrow HPCs (Yang et al., 2014). However, other studies have also shown that the effect of promoting hematopoiesis was not the best, as the compatibility ratio of AR and ASR was 5:1, and all combinations had a synergistic effect on promoting hematopoietic function recovery, as the ratio ranges from 1:5 to 5:1 (Shi et al., 2012). It was suggested that AR and ASR could play a better role in promoting hematopoiesis when they were combined in a certain proportion range. Studies have shown that saponins of astragaloside III and AST and flavonoids of CAL and FRM from AR and FRA, an organic acid from ASR, are the most abundant ingredients in DBT (Zhang et al., 2012).

Caco-2 cell research showed that the permeability of monolayer membrane in caco-2 cells and the absorption of AST, CAL, and FRM could improve in the presence of FRA (Zheng et al., 2012). However, the main chemical components in the volatile oil of the ASR are artemisia ligustilide, a negative regulation, which inhibits the biological effect of DBT. In the presence of ligustilide, the amount of AST, CAL, FRM, and total polysaccharides extracted from AR was decreased (Zheng et al., 2010).

Our studies also showed that the 1:1 compatibility of AR-ASR can promote the dissolution and absorption of main active components AST, CAL, CLD, FRM, and FRA in isolated small intestine of rats (Li et al., 2017). Therefore, according to the literature reports and our study, we chose the compatibility of AR-ASR with 1:1, which has the strongest hematopoietic effect, and selected AST, CAL, CLD, FRM, and FRA as the main effective components for research. The content of five active components in the compatibility of AR-ASR (1:1) was firstly determined. Then, we selected the best compatibility of AR-ASR (1:1) for promoting hematopoiesis and determined the proportion of the five components’ compatibility (FRA : FRM:AST : CAL:CLG = 23:11:24:16:56) based on content assay of the five main active components. Aging of HSCs can be caused by body aging or the action of chemical, radiation, and other factors, thus leading to abnormal self-renewal ability and differentiation function of HSCs and block of cell proliferation cycle, which is the main cause of low hematopoietic function (Florian et al., 2012).Therefore, on the basis of studying the compatibility of the main components of AR-ASR, we studied the effect of the compatibility of the five active components on the proliferation of HSCs with aging model, so as to reveal the potential mechanism.

RETRACTED

CTX has cytotoxicity, which can damage bone marrow hematopoietic stem/progenitor cells and inhibit bone marrow hematopoietic function, kills peripheral blood cells, and reduces blood cell count. After drug withdrawal, myelosuppression induced by cyclophosphamide can be recovered by itself (Li et al., 2017). In our previous studies, we found that RBCs, WBCs, PLTs, and Hb in peripheral blood gradually decreased and fell to the lowest level at 5–6 days after the start of CTX injection, and recovered to nearly normal level at the seventh day after the stop of CTX injection. Therefore, it was determined that the hematopoietic function of CTX-induced myelosuppression mice should be assayed on the sixth day after the CTX injection. The results indicated that both AR-ASR compatibility (1:1) and the combination of the five active components could increase the number of RBCs, WBCs, PLTs, and content of Hb in peripheral blood and add to the area of bone marrow hematopoietic tissue. The increase in AR-ASR compatibility (1:1) had the same effect as the five active components combination, which showed that the five active components are the main pharmacodynamic substances of AR-ASR compatibility to promote hematopoiesis. Further analysis showed that the five active components could increase the number of RBCs and Hb content in peripheral blood, which suggested that five active components are the main active components in increasing peripheral blood RBCs. FRA could increase the number of WBCs, which suggested that FRA is the main pharmacodynamic substance to increase peripheral blood WBCs. With regard to PLTs, the results showed that only FRA and AST could increase the number of PLTs in peripheral blood, which indicated that FRA and AST are the main pharmacodynamic substances to increase peripheral blood PLTs. Bone marrow morphology studies showed that only FRA could increase the bone marrow hematopoietic tissue area. It suggested that FRA is the main pharmacodynamic substance to inhibit the atrophy of bone marrow hematopoietic tissue induced by CTX. It also suggested that the five active components of AR-ASR could increase the different blood cells in the peripheral blood in bone marrow suppression mice, and the five active components might be the main pharmacodynamic components to promote hematopoiesis, and the combination of the five active components could enhance its hematopoietic effect.

RETRACTED

On the basis of confirming the main components of AR-ASR and their compatibility to promote hematopoiesis, we studied the possible mechanism from HGF and HPC proliferation in mice. Hemocytogenesis of mammals occurs in the complex hematopoietic environment of the marrow cavity. Formal ingredients were derived from the proliferation and differentiation of HSCs and HPCs. However, all kinds of mature blood cells (except lymphocytes) live from a few hours to a few days. BMNCs adapted this property and could renew and proliferate, in a way that continuously generates RBCs, WBCs, and PLTs, so as to maintain a dynamic balance of blood physical components, thereby maintaining the survival and proliferation of each hematopoietic lineage and promoting the differentiation of HGFs and their corresponding receptors (Watowich et al., 1996). HGFs mainly include EPO, TPO, and CSF, which could affect many aspects of the hematopoietic process, thereby regulating the survival, growth, and development of primitive blood cells. This study provides further evidence that AR-ASR compatibility (1:1) and the combination of five active components could increase serum EPO, TPO, and GM-CSF, and both had similar effects. However, only FRA, CAL, and CLG increased the content of serum EPO, which suggested they may be the main substances that promote the synthesis and secretion of EPO. FRA and CAL increased serum GM-CSF content, suggesting that they may be the main pharmacodynamic substances to promote GM-CSF synthesis and secretion. FRA, FRM, AST, CAL, and CLG all increased serum TPO content, suggesting that all five active components may promote the synthesis and secretion of TPO.

HPCs are primary myeloid nucleated cells with proliferative capacity, which can generate corresponding progenitor cell colonies stimulated by different CSFs. There are three main types of HPCs: first, granulocyte-macrophage HPCs are a cell colony that must be formed under the action of GM-CSF, and they are called CFU-GM. Second, megakaryocyte HPCs are a cell colony that must be formed under the action of TPO and are called CFU-MK. Third, erythroid HPCs are a cell colony that can be formed only under the action of EPO, and they are called CFU-E and BFU-E (Gallicchio et al., 1987). Therefore, detecting the proliferation of HPCs *in vitro* could reflect the hematopoietic capacity of the body. Studies have shown that either the DBT (AR : ASR = 5:1) or the combination of AR-ASR (AR : ASR = 1:1) could promote HPC proliferation in animals with myelosuppression (Yan et al., 2014; Li et al., 2017). This study indicated that AR-ASR compatibility (1:1) and the combination of five active components could increase the colonies of CFU-GM, CFU-MK, CFU-E, and BFU-E, and both had similar effects. The study also suggested that these two could promote HSC proliferation in mice with suppressed bone marrow hematopoietic function, and they had similar effects. It can be seen that the pharmacophore in AR-ASR promoted the proliferation of HPCs by promoting multiple cells to synthesize and secrete HGFs. All active components (FRA, FRM, AST, CAL, CLG) could promote the proliferation of CFU-E and BFU-E, which suggested that five active components may be the main pharmacodynamic substances to promote the proliferation of erythroid progenitor cells. FRA, CAL, and CLG could promote the proliferation of CFU-MK, which suggested that the three active components may be the main pharmacophores to promote the proliferation of megakaryocytes. FRA, FRM, CAL, and CLG could promote the proliferation of CFU-GM, which suggested that the four active components may be the main pharmacophores to promote the proliferation of granulocyte-macrophage progenitor cells.

RETRACTED

From the above experiments in mice, we have proved that the five main components of AR-ASR could promote hematopoiesis. Therefore, we further studied the effects of five main components on the proliferation of aging HSCs *in vitro*. HSCs are the seed cells of the hematopoietic system of the body, with strong potential for multidirectional differentiation and self-renewal (Eaves, 2015). Aging, radiation, and anti-tumor chemotherapy drugs can cause the aging of bone marrow HSCs, resulting in low proliferation and differentiation function, thus reducing hematopoietic function (Nijnik et al., 2007). The significant features of HSCs aging include reduced self-renewal ability, abnormal differentiation function, cell proliferation cycle retardation, and obviously delayed proliferation response (Dykstra et al., 2011). Various emergency factors such as chemotherapy, radiotherapy, and reactive oxygen species are important causes of HSC aging and cell cycle cessation. It is believed that the formation of HSCs is related to a variety of mechanisms, among which the p53/p21 signaling pathway plays an important role. In emergency conditions (such as DNA damage, hypoxia, and infection), p53 activation plays an important role in protecting cell survival. Activation of p53 by damaged DNA leads to high expression of p21, which can effectively inhibit CDK and cause cell cycle cessation. Meanwhile, p53 activation and p21 high expression induced by upregulation of p14 ARF or nutlin-3 could lead to fibroblast aging (Villalonga-Planells et al., 2011).

t-BHP is an inducer of oxidative stress, which can induce excessive ROS production in cells, leading to cell damage, necrosis, and apoptosis (Zhao et al., 2017). Studies have shown that t-BHP could reduce self-renewal and multidirectional differentiation potential of HSCs/HPCs. The number of HPC mixed colonies (CFU-mix) decreased and irreversible stagnation in G1 phase, the positive rate of SA-beta-Gal staining increased, and characteristic changes of senescent cells appeared, which suggest that t-BHP could construct an *in vitro* senescence model of Sca-1^+^HSC/HPC (Zhou et al., 2011). SA-β-Gal staining is an important biological marker for cell senescence identification. Only senescent cells can be stained, whereas pre-senescence cells, dormant cells, and tumor cells cannot, and the results are reliable without interferences by other hybrid cells (Zhou et al., 2011). Therefore, the aging model of HSCs induced by t-BHP was further adopted to study the effects of five components of AR-ASR on the proliferation of aging HSCs. This study showed that FRA (the active component of ASR), AST, and FRM (the active components of AR) could significantly promote the proliferation of aging HSCs in a dose-dependent manner. CAL and CLG had no significant effect on promoting the proliferation of aging HSCs when used alone, but orthogonal experiments showed that CAL and CLG combined with FRA, AST, and FRM could significantly promote the proliferation of aging HSCs. In addition, CAL, CLD, FRA, AST, and FRM showed synergistic effects in promoting cell proliferation and inhibiting cell senescence. Experiments also show that FRA, AST, and FRM had a strong effect on accelerating the transformation of the aging HSC cell cycle, reducing the number of cells in the stationary phase, and increasing the number of cells in the proliferative phase. In addition, CAL and CLG had a weak role in promoting cell cycle transformation. The effect of the five active components on promoting cell cycle transformation was significantly stronger than that of the single active components. The effect of AR-ASR compatibility (AR : ASR = 1:1) and the combination of five active components were quite high in promoting the proliferation of aging HSCs and reducing the positive rate of aging cells. It was further verified that five active components had the same effect as that of AR-ASR compatibility (AR : ASR = 1:1). Five active components were the main effective substances from AR and ASR to promote hematopoiesis.

RETRACTED

Results of Western blot showed that FRA, AST, and FRM could promote the expression of cyclin D1 and CDK4 proteins in aging HSCs; CAL and CLG also had a weak role. The expression of cyclin D1 and CDK4 protein as five active components combination was significantly higher than that of the five active components alone. Our study showed that the combination of the five active components could promote the expression of cyclin D1 and CDK4 proteins in aging HSCs. Cyclin D1 and cyclin E play key roles in regulating the cell cycle G0/G1 and G1/S transformation, and they determine whether cells are transformed from the nonproliferative state to the proliferative state. Cyclin D1 is a specific protein of cell cycle G1. Cyclin D1 binds and activates cyclin-dependent kinases CDK4 and CDK6 and then phosphorylates its downstream target proteins and shortens the cell cycle by accelerating the process of the G1 phase (Coqueret, 2002). CDK regulates cell cycle progression in a positive way by binding to cyclin. Different cyclins recognize and combine with different CDKs to form different cyclin–CDK complexes. The combination of CDK4 and cyclin D1 can cause the retinoblastoma tumour suppressor (Rb) protein to lose its blocking effect on cell cycle by phosphorylating the Rb protein and realizing the effect of promoting and transforming the cell cycle (Pines, 1995). Therefore, it is speculated that the combination of AR and ASR may promote the proliferation of aging HSCs, which may promote the expression of cyclin D1 and CDK4 proteins and consequently shorten the cell cycle and accelerate the process of the cell cycle.

## Conclusion

To summarize, animal experiments (*in vivo*) showed that AR-ASR compatibility (AR : ASR = 1:1) and five active components could improve the hematopoietic function of bone marrow and inhibit the hematopoietic function in mice, improve the content of peripheral hemogram and HGFs, and promote the proliferation of HPCs. Cell experiments (*in vitro*) showed that the combination of AR-ASR (AR : ASR = 1:1) and its active components could improve the aging of HSCs, shorten the cell cycle, and promote HSC proliferation. The combination of the five active components had a synergistic effect, which suggested that different active components acted on different hematopoietic processes, thereby promoting the proliferation and differentiation of HSCs/HPCs and playing an enhanced role in promoting hematopoiesis.

However, due to the complex composition of TCM and the complex hematopoietic regulatory mechanism, which link do these main active components act on? The mechanism of promoting the proliferation and differentiation of HSCs is still unclear and needs further study in the future.

## Data Availability

The raw data supporting the conclusions of this manuscript will be made available by the authors, without undue reservation, to any qualified researcher.

## Ethics Statement

This study was carried out in accordance with the recommendations of the ethical standards of Guide for the Care and Use of Laboratory Animals (No. 86-23; NIH Publications, 1996) and the protocol was approved by the Animal Ethics Committee of Hunan University of Chinese Medicine (approval No. 43004700005819, date: April 25, 2014).

RETRACTED

## Author Contributions

WZ, X-PH, and C-QD designed the research project. J-HZ and HX performed the experiment. WZ and X-DL analyzed the data. J-HZ and HX contributed the reagents and materials. WZ and X-QD wrote and modified the manuscript.

## Funding

This work was supported by the grants from the National Nature Science Foundation of China (No.81473581, No.81774032, No.81874406), Hunan Natural Science Foundation (No.2016JJ4069), and Hunan Education Department open Foundation (No.15k089).

## Conflict of Interest Statement

The authors declare that the research was conducted in the absence of any commercial or financial relationships that could be construed as a potential conflict of interest.
